RETRACTED

# Exploration on the Role of Transformational Leadership Linkage Psychological Empowerment in Stimulating Employees' Innovation Behavior in an Uncertain Environment: Based on Entrepreneurship Perspective

**DOI:** 10.1155/2022/9259180

**Published:** 2022-09-19

**Authors:** Xiaoying Wei, Ying He

**Affiliations:** ^1^School of Business, Nanjing University, Nanjing City 210093, China; ^2^School of Business Administration, Baise University, Baise City 533000, China

## Abstract

Employee Innovative Behavior (EIB) in a stable environment is often based on the company's planned policy orientation and has higher innovation performance under the transactional leadership behavior characterized by task orientation. In an uncertain environment, transformational corporate leadership behaviors will stimulate EIB. The essence of entrepreneurship is innovation. Enterprises provide employees with spiritual support through entrepreneurship, which can generate more effective long-term incentives for employees. From the perspective of entrepreneurship, based on the Uncertainty-Identity Theory (UIT), through the analysis of 287 pairs of valid sample data from 7 companies, it is found that Environmental Uncertainty (EU) has a positive moderating effect on the relationship between Transformational Leadership (TL) and Psychological Empowerment (PE). PE positively promotes EIB. The indirect effect size of PE is 0.2221, 0.3495, and 0.4450 from low to high, respectively. It is inferred that the interaction between TL and EU can positively promote EIB through the mediating effect of PE. The research conclusions expand the boundary conditions of the relationship between TL and EIB and innovatively provide theoretical guidance for the management of EIB from the perspective of entrepreneurship in an uncertain environment.

## 1. Introduction

In 2018, the US Department of Commerce announced a seven-year ban on ZTE [1], followed by sanctions on Huawei for chip supply, restricting the supply of chips based on US technology or patents to Huawei. A report by China Everbright Securities shows that many Chinese companies that rely on US core technology and proprietary chips and other accessories are still in US hands [2]. In the context of the new normal of the economy, the traditional production model is difficult to meet the changing times and consumer demands. As an important main body of the market economy, enterprises bear the heavy responsibility of continuous innovation. The continuous intervention and sanctions by the US on the supply of related technical products and accessories have pushed Chinese enterprises to the outlet of independent innovation, which once again shows that only relying on independent innovation can promote the survival and development of enterprises in an uncertain environment. And enterprises urgently need to find breakthroughs through innovation [3]. The innovation inherent in entrepreneurship itself makes it play a pivotal role in enterprise operation management and Employee Innovative Behavior (EIB) and has a positive impact on EIB and enterprise performance.

RETRACTED

Employees are the main foundation of enterprise innovation and change, and the technological innovation and development of an organization cannot be separated from the occurrence of individual innovative behaviors [4]. The innovative behavior of employees is the behavior they take after evaluating the environmental factors. In a relatively stable and orderly environment, employees have a high degree of predictability and control over the results of innovative behaviors, and the cost of trial and error in the process of innovative behaviors is relatively low. Under this condition, EIB is often based on the enterprise's planned policy orientation and has higher innovation performance under the transactional leadership behavior characterized by task orientation [5]. However, the rapid development of emerging technologies such as big data, cloud computing, biotechnology, and artificial intelligence has aggravated the dynamic uncertainty of the environment, coupled with the influence of natural and social factors. For example, the global spread of COVID-19 has disrupted the global industrial chain and even changed the world pattern [6].

People are facing unprecedented changes in the times. How to deal with the challenge of this uncertainty is a problem that all enterprises should think about at present. Facts have proved that only change and innovation can enable enterprises to survive and develop in an uncertain environment. However, in the face of high internal and external Environmental Uncertainty (EU), how can companies effectively stimulate EIB? This is not only an urgent problem to be solved in reality but also a problem to be explored in research.

## 2. Literature Review

Although there are many studies on how to promote EIB, the issue of how to stimulate EIB in an uncertain environment is still lacking in-depth discussions. Bos believes that [7], when the individual's perception of uncertainty is high, due to the lack of predictability and control over the environment, it will cause strong anxiety and unease, which will affect the individual's cognition, emotion, and behavior. To reduce this sense of uncertainty, employees desire fair information and perceptions of organizational justice. As a representative of the formal power of the organization, corporate leadership is the configurator and controller of organizational resources. Corporate leadership behavior and leadership style can convey organizational information to employees through organizational behavior, help employees balance uncertainty perception, and thus affect employee cognition and behavior. Therefore, under the perception of high uncertainty, the organization needs to use the power of leadership to create an organizational atmosphere that is conducive to stimulating EIB [8]. Among many leadership styles, Transformational Leadership (TL) is considered to be a leadership behavior that is more dynamic and capable of controlling uncertain situations. It is better at turning uncertain environments into opportunities and challenges. Through the influence of vision blueprints and moral appeal, employees can internalize organizational goals, create a unified value organizational culture, and arouse subordinates' sense of identity with the organization [9].

RETRACTED

British psychologist Hogg [10] put forward the Uncertainty-Identity Theory (UIT) in 2000 based on social identity theory and self-classification theory. The theory describes how identity-related uncertainty motivates people to identify with social groups, reducing uncertainty through group identification and categorization of self and others. Specifically, when employees perceive EU as high and for a long time, they will strengthen their identification with organizations with similar values to their own, thereby enhancing their sense of belonging and indirectly alleviating uncertainty. In a highly uncertain environment, TL can form a unified organizational culture of organizational goals and values within the organization, which in turn can enhance employees' identification with the organization and arouse employees to obtain a sense of belonging to the organization [11]. Meanwhile, transformational leaders value the individual needs of their employees, empower them appropriately, and provide them with individualized support [12]. Driven by the sense of ownership and based on the viewpoint of social exchange theory, TL behaviors can effectively motivate employees to practice innovative behaviors that are beneficial to organizational development, improve innovative performance, and reward the organization. TL provides employees with a supportive atmosphere for organizational innovation, which will further promote employees to transform their responsibility and self-efficacy into innovative behaviors that are beneficial to organizational development.

Therefore, this paper attempts to explore the role of psychological empowerment (PE) such as employees' sense of belonging, work significance and influence, and self-efficacy from the perspective of entrepreneurship. The mechanism of TL based on entrepreneurship to stimulate EIB in an uncertain environment is revealed. The interaction between TL and EU is explored. The process of stimulating EIB through employees' PE is expected to provide theoretical guidance for enterprise managers to stimulate EIB management based on the perspective of entrepreneurship in an uncertain environment and also expand the boundary conditions of the relationship between TL and EIB. The research innovation point is to study the scheme of managing EIB based on entrepreneurship in an uncertain environment.

RETRACTED

## 3. Theoretical Basis and Research Hypothesis

### 3.1. Entrepreneurship Theory

Entrepreneurship is the entrepreneurs' ability to effectively utilize the existing ESE resources to create output, leading the company to exchange smaller investments for a larger income. In a certain sense, entrepreneurship is realized as improving ESEs' performance through Resource Utilization Efficiency (RUE) [13]. The individual characteristics of entrepreneurs affect the company value by influencing the company's strategic Decision-Making (DM). Due to the complexity of the external environment, entrepreneurship leads the determination of the values and existing cognitive structure of the top management team, thereby improving the management's ability to draw on resources and make strategic decisions and IB to enhance ESE performance. Therefore, entrepreneurship plays a key role in the quality and SD of ESEs. As the engine of ESE development, entrepreneurship is an extremely scarce resource and important soft power in society.

On the other hand, entrepreneurship is a part of ESE culture. Its essence is change and innovation. Entrepreneurship improves the organizational structure through change and obtains profits, creates material wealth, improves ESE's competitiveness, and promotes social progress through the IB of managers and employees at all levels. Based on the leadership style of entrepreneurs, it can be divided into TL style and transactional leadership style. Of these, the transactional style will weaken the positive impact of entrepreneurship on Corporate Social Responsibility (CSR), while the TL style can significantly and positively affect corporate entrepreneurship [14]. Under the economic transformation of the current international environment, it is of great practical significance to explore the economic effects of high-level behavior of ESEs under the guidance of entrepreneurship and the impact mechanism on EIB [15]. By studying entrepreneurship theory, it is possible to more effectively study the impact of TL on ESEs. This paper is aimed at analyzing the mechanism of the relationship between TL and EIB in an EU from the perspective of entrepreneurship.

RETRACTED

### 3.2. Transformational Leadership Beneficial to Stimulate Employee Innovative Behavior

In a relatively static, stable, and orderly environment, employees usually carry out innovation activities under the planned policy guidance of the organization. Their IB follows certain organizational practices and rules, guaranteed by a relatively stable organizational system. The TAE cost of EIB is relatively low. Task-oriented transactional leadership behavior can effectively improve employees' innovation performance. However, given the rapidly changing EU, without predictability and controllability of the environment, individuals lose their sense of security, which will affect individual cognition and self-consciousness, thus affecting the generation of IB [16]. In the context of strong internal and external uncertainty perception, it is necessary to create an organizational atmosphere conducive to employees' innovation and creativity by influencing specific leadership behavior to stimulate EIB.

As two important concepts in leadership theory, TL is significantly different from transactional leadership. Transactional leadership pays attention to standards and norms, emphasizes employee loyalty, and likes a stable and fixed working environment. In contrast, TL leaders are considered to like challenges and risks, be good at capturing opportunities brought by environmental changes, make full use of favorable conditions and factors, and combine power to mobilize employees' psychological motivation for innovation and change; meanwhile, they try their best to tap employees' potential, encourage employees to participate in change and innovation, rethink new situations rationally, and work with innovative methods; moreover, TL enables organizations to adjust their operation mode against the rapidly changing environment to achieve higher organizational goals. For instance, Burns [17] contended that TL was to pursue higher organizational goals, stimulate employees' high-level needs through the psychological level, try to motivate subordinates, pay attention to instilling the values of respect and honor in employees, and emphasize the motivation of authorization and endogenous motivation; in this way, higher organizational goals could be obtained. On the other hand, TL pays attention to employees' DC participation and provides personalized resource support to create a cultural atmosphere and Fault-Tolerant (FT) environment for organizational innovation support, thereby reducing the risk of TAE from employees' innovation failure. Additionally, TL stresses the construction of unified ESE values and culture, influencing subordinates from high-level psychological needs, internalizing organizational goals, and strengthening subordinates with higher morale and motivation. Further, in an EU, TL can enhance employees' recognition of the organization, arouse employees' organizational SOE, and stimulate their organizational SoR and SoO. Based on the perspective of mutual benefit and win-win, employees will more actively use autonomy and organizational resources to practice IB for organizational development. When the environment changes and presents dynamic and complex characteristics, TL turns the changing and EU into opportunities and challenges, depict higher organizational goals, and vision blueprints to employees, and employees, based on high-level psychological needs, in the context of high-expectation tasks brought about by changes inside and outside the organization, are more likely to find new problems in organizational development and actively explore feasible solutions, to contribute to ESE performance and personal growth. Based on the above analysis, this paper puts forward the following hypotheses:

H1: In the EU, TL positively promotes EIB.

RETRACTED

### 3.3. Influence of PE (Psychological Empowerment) on Employee Innovative Behavior in Environmental Uncertainty

PM refers to the complex four cognitive psychological states experienced by authorized individuals: work significance, SE, autonomy, and work impact [18]. In other terms, PM can also be defined as a kind of psychological experience with a vision of job prospects and a sense of internal control of SE [19]. If employees have sufficient PE (Psychological Empowerment) perception, it shows that the organizational work requirements match the values and beliefs of employees. In other words, employees believe that they can affect the organization's strategy and development direction. They have obtained full autonomy and have enough ability and skills to complete the organizational tasks. In particular, EIB is driven by the endogenous motivation of high-level psychological needs; PE is deemed one of the primary factors to promote employees' endogenous motivation [20]. In an EU, due to the increased risk from TAE, EIB depends more on the employees' organizational SoB, SoO, and SoR, the work autonomy of employees' endogenous motivation, and an organizational FT atmosphere [21]. PE can improve employees' organizational SoB; work autonomy; their SoO, SoR, and SE; and the perception of organizational FT atmosphere [22]. Driven by the SoO, SoR, and SE, employees are more active in exploring innovation, trying to find possible solutions to problems, and improving work efficiency and organizational performance to repay the organization, which is more likely to produce organization-beneficial IB. Thereupon, the following hypothesis is proposed:

H2: In the EU, PE has a positive impact on EIB.

RETRACTED

### 3.4. The Mediating Effect of Psychological Empowerment on the Relationship between Transformational Leadership and Employee Innovative Behavior in an Environmental Uncertainty

EIB is an organizational citizenship behavior with strong autonomy, which is driven by employees' high-level internal psychological needs [23]. In an EU, employees with organizational SoB, SoO, and SoR will actively seek innovative ways to participate in organizational change and improve organizational operation, while TL leaders advocate giving employees work resources and appropriate authorization, strengthening employees' work autonomy and DC participation, and emphasizing the internalization of organizational objectives. Therefore, the behavioral characteristics of TL can enhance employees' PE, promote employees' endogenous motivation, and then stimulate EIB. Under the influence of TL behavior, based on the organizational SoB and SoR, employees are inspired to repay the organization from the bottom of their hearts so as to practice the organization-beneficial IB; additionally, in the EU, TL leaders turn uncertainty into development opportunities, put forward high-performance expectations for employees, strive to stimulate employees' high-level needs, help employees recognize their work significance, and pay attention to intellectual stimulation and personalized care, thus improving employees' SE. From the perspective of social cognition, employees perceive high work expectations and significance and expect to achieve their work expectations in this environment based on high SE and organizational support. This psychological experience will urge employees to implement innovative activities conducive to organizational development to obtain expected results. Thereupon, the following hypothesis is proposed:

H3: In an EU, PE plays an intermediary role between TL and EIB.

### 3.5. Regulation of Environmental Uncertainty

EU is often used to describe the situation of the organizational environment and the sense of uncertainty individuals perceive due to their lack of access to key organizational information. Likewise, BOS et al. [7] suggested that the EU was a dynamic, complex, and uncontrollable or predictable environment faced by the organization. This environment might bring great threats and risks to the organization, causing anxiousness and uneasiness among the organization members and thus affecting their attitude and behavior. Employees under a high degree and long-term internal and external organizational uncertainty, according to the viewpoint of UIT [10], would form the self-belonging needs of “who am I” and “how should I do” to reduce the uncertainty and classify themselves with others as group members, to provide both parties with an effective social identity. This classification process can effectively reduce self-uncertainty, and the more an organizational member is in a high uncertainty environment, the more likely the member is to identify with high entity groups or organizations similar to their own values, and they will be committed to joining them, hence recreating them or transforming the existing groups into more entity. This can be well illustrated by a quote by Dewey, a pragmatist philosopher [24]: in a dangerous world, in the absence of real certainty, people will cultivate all kinds of things that can make them feel certain of safety.

RETRACTED

The TL leaders are suitable for turning the EU into opportunities and challenges. For example, under environmental changes, they encourage employees to use modern technologies and methods to solve new problems and difficulties, unite with higher passion and higher morale, draw a beautiful vision blueprint for subordinates, influence subordinates through the psychological level, internalize organizational goals, and form unified organizational cultural values. When facing high EU, people are more eager to organize their own identity. They tend to identify with entity organizations similar to their own values. Under the high EU, TL can better promote employees to further identify with the organization. TL leaders' high expectations and authorization help employees recognize their work significance better. It also enhances employees' work autonomy and SE. Previous studies have shown that a high degree of self-uncertainty drives individuals to identify with and support radical group organizations. So far, studies have corroborated that [25] uncertainty will strengthen identity, employees' self-uncertainty will surpass self-improvement, and employees need more positive and respected leadership behaviors to tolerate and reduce uncertainty when they have high uncertainty perception. Therefore, the higher the EU is, the more effective the TL behavior can enhance the PE of organizational members. Conversely, in the context of low EU, due to the stability of the situation, ESEs usually maintain the original organizational practices, employees follow the original rules and inertial thinking, and employees' organizational ownership needs for self-classification and seeking effective identity are relatively weak. At this time, the impact of TL behavior on employees' higher psychological needs is relatively low. Due to the lack of new opportunities and high work challenges, employees are less aware of leaders' high expectations and authorization support, and their sense of work significance and importance is also low. Therefore, when the degree of EU is low, the impact of TL on employees' PE is relatively weak. Accordingly, the following hypothesis is proposed:

H4: EU positively regulates the relationship between TL and PE.

RETRACTED

Based on the above analysis, this section constructs the following research model, as illustrated in Figure 1.

## 4. Research Design

### 4.1. Sample and Data Collection

In this study, data is collected by questionnaire survey (QS). The samples are from seven high-tech enterprises in Guangxi, Guangdong, Jiangxi, and Zhejiang. The respondents are mainly employees and their superiors in the Research and Development (R&D) and Service Departments because the work of these departments has high flexibility and autonomy. The data is collected using a leader-employee paired sample. In order to reduce homologous variance and improve data quality, this study selects two time periods to collect data. The first period is mainly concentrated in December 2020. The questionnaire is filled out by employees with demographic characteristic variables such as gender, age, working years, and education level, as well as TL and PE.

The second questionnaire is issued and filled out in March 2021. The employees who completed the questionnaire for the first time filled out the EU variable option, and the subordinate superior leaders were matched with the employees who filled out the EIB variable option. The questionnaire is issued and collected using entrusted investigation, and timely contact and communication are conducted by telephone. First, the researchers communicate with the Human Resources (HR) of the company concerned about the survey, stating that the survey data is used only for academic research. Then, the enterprise HR department designates the person in charge of screening out the qualified department staff and their superiors and explains the questionnaire filling requirements. The QS is distributed to them to fill in after recycling.

The selected sample is paired with employees and their immediate superiors. Finally, by sorting and screening the recovered questionnaires in two stages, a total of 287 pairs of valid paired questionnaires are finally determined. Among the respondents, male employees accounted for 66.3% and employees with a bachelor's degree or above accounted for 64.2%. The average age of the surveyed employees is 32.3 years, mainly young people. 72.7% have worked for less than 5 years, and most employees have shorter working years. In the leadership sample, 58.2% of them have worked for more than 5 years.

RETRACTED

### 4.2. Variable Measurement

The measurement indicators include TL, PE, EU, and EIB. In order to better complete the measurement, mature measurement scales are adopted in the academic world. In order to ensure the validity of the use of the scale and the accuracy of the meaning of the items, a total of 2 management experts and professionals are invited to review the scale. Except for the control variable, all scales are 5-point Likert scales, with 1 for “strongly disagree,” 3 for “uncertain,” and 5 for “strongly agree.” Figure 2 shows the overall research framework.

#### 4.2.1. TL

The TL QS suitable for China's national conditions prepared by Wang et al. [26] is chosen combined with China's situation, including four dimensions and 14 items: core TL behavior, high-performance expectation, individual support, and intelligence stimulation, in which *α* = 0.95. Many representative topics are involved, such as “leaders clearly express the common vision,” “leaders urge us to accept the common goal of the team,” “leaders will consider our feelings before action,” and “leaders encourage us to think about old problems in new ways.”

#### 4.2.2. PE

The Chinese version of the QS suitable for the Chinese situation prepared by Spreitzer [19] and revised by Li et al. [27] is adopted. There are 12 questions in total, including 4 dimensions, in which *α* = 0.81. Representative questions involve “what I do at work is very meaningful to me personally,” “I can decide how to start my work,” and “I am very confident in my ability to complete my work.”

#### 4.2.3. EIB

It adopts the Chinese version of the scale translated and revised by Liu et al. [28], containing nine items with *α* = 0.87. Typical questions entail “the employee often actively searches for new working methods, technologies, or tools” and “the employee often turns new ideas into useful practice.”

#### 4.2.4. EU

The scale of the De Hoogh [29] version is adopted and modified in combination with the actual situation, including three items (example, the working environment of the department is full of changes), in which *α* = 0.82.

#### 4.2.5. Control Variables

Based on the existing research [22], this paper sets employee gender, age, educational level, and working seniority as control variables.

## 5. Data Analysis and Results

### 5.1. Confirmatory Factor Analysis (CFA)

To test the discriminant validity between TL, PE, EU, and EIB, Amos22 0 CFA is performed on four variables, and the results are illustrated in Table 1.

RETRACTED

Compared with the three-factor, two-factor, and single-factor models, the four-factor model has better validity (*χ*^2^/df, GFI = 0.869, NFI = 0.885, TLI = 0.970, CFI = 0.973, and RMSEA = 0.031). Thus, the four variables in the model have good discriminant validity.

### 5.2. Descriptive Statistics and Correlation Analysis

Table 2 presents the descriptive statistical analysis results such as the mean value and standard deviation of each variable, as well as the correlation coefficient matrix between the variables. Table 2 shows that there is a significant positive correlation between TL and EIB (*r* = 0.57, *p* < 0.01). Therefore, this data result indicates that Hypothesis 1, Hypothesis 2, and Hypothesis 3 have been preliminarily verified.

### 5.3. Hypothesis Test

#### 5.3.1. Mediating Effect Test

The hierarchical regression method recommended by Baron and Kenny [30] is used to test the mediation effect through the software SPSS22.0, and the Boostrap method recommended by Preacher and Hayes [31] and Chen et al. [32] is inserted into SPSS to further test the moderated mediation effect. The models of PE and EIB under different mediation effects are verified, respectively, as shown in Table 3. The model contains 6 models, and models 1-3 represent various factors under the influence of variable PE. Models 4-6 represent the various factors under the influence of the variable EIB.

First, the main effect relationship between the independent variable and the dependent variable is tested. Model 4 in Table 3 shows that after controlling for gender, age, education, and working years, TL has a significant positive impact on EIB (*β* = 0.471, *p* < 0.001), and Hypothesis 1 is verified. Second, the relationship between independent variables and mediator variables is verified. Model 1 in Table 3 indicates that TL has a significant positive impact on employees' PE (*β* = 0.599, *p* < 0.001). Model 5 suggests that PE has a significant positive impact on EIB (*β* = 0.601, *p* < 0.001), and Hypotheses 2 and 3 are verified. Finally, whether the mediating variable is completely mediating is verified, and the independent variable and mediating variable are added into Model 6; the mediating variable PE positively affects EIB (*β* = 0.500, *p* < 0.001). Meanwhile, TL has not disappeared on EIB, and there is still a significant positive impact, but the effect is significantly weakened (*β* = 0.191, *p* < 0.001), which proves that PE plays a partial mediating role between TL and EIB in an uncertain environment.

In order to further test the intermediary role of psychological empowerment between TL and EIB, this section refers to the methods recommended by Preacher and Hayes and Chen et al. and inserts the Process plug-in into SPSS for Bootstrap (model 4) to test. Then, it sets the random sample to 5,000 times and the confidence level to 95%.

RETRACTED

The results are shown in Table 4 and Figure 3. At the 95% confidence level, the confidence interval does not include 0 [0.2955, 0.5188], and the mediating effect of PE is significant. After controlling the indirect effect of PE, the direct effect between TL and EIB is also significant, and the 95% confidence interval does not include 0 [0.0629, 0.3870]. It further verifies that PE plays a partial mediating role between TL and EIB.

#### 5.3.2. Test of Regulatory Effect

In order to test the moderating effect of EU between TL and PE, according to the hierarchical regression method, the variables are first centralized, and then, the product items are constructed. The results are shown in Table 3 and Figure 4. According to Model 3, the interaction between TL and EU has a significant positive impact on employees' PE (*β* = 0.363, *p* < 0.01), and Hypothesis 4 is verified.

In order to verify the mediated regulatory effect, this section refers to the method recommended by Preacher and Hayes [31] and Chen et al. [32] and inserts the Process plug-in into SPSS for Bootstrap (model 8) to test. Five thousand samples are randomly selected, and the CI is 95%. The results are revealed in Table 5. Under the EU, PE mediates the relationship between TL and EIB, and under the adjustment of low-, medium-, and high-level EU, the mediating effect of PE is significant, and the CIs are [0.7660 and 0.3690], [0.2472, 0.4600], and [0.3240, 0.5694], respectively, all of which do not contain 0. Meanwhile, the indirect effect values from low to high are 0.2221, 0.3495, and 0.4450, respectively. The results corroborate that the higher the EU is, the stronger the mediating role of PE between TL and EIB is.

In order to intuitively show the moderating effect of EU on PE, this paper refers to the method recommended by Cohen et al. [33] and draws a difference map of the response of TL to PE based on EU above the mean and below the mean one standard deviation level, as shown in Figure 5.

## 6. Discussion of the Results and Analysis of Implications

### 6.1. Discussion of the Results

Based on a questionnaire survey of 287 paired sample data of 7 enterprises, the mechanism and boundary conditions of TL are discussed to stimulate EIB in an uncertain environment and draw the following conclusions:

1. In an uncertain environment, TL has a significant positive impact on EIB. This research conclusion is an extension of the previous research results of scholars [34, 35], which further confirms that TL can promote EIB even in uncertain situations. When the external environment is dynamic and uncertain, TL can influence subordinates at the psychological level, transform uncertainty into opportunities and challenges, unite organizational members with higher morale, and encourage employees to try to deal with future uncertainty in different ways of working and behavior when facing new situations. TL creates an organizational atmosphere that encourages and supports innovation, creates an inclusive organizational fault-tolerant environment, and further promotes the generation of EIB
2. PE partially mediates the impact of TL on EIB. This research conclusion expands the boundary conditions of the research results of previous scholars [22, 36] and confirms that TL can promote and stimulate EIB through the mediating role of PE in an uncertain environment. Bass [37] believed that TL behavior is conducive to improving employees' self-efficacy and helping employees realize the importance of their tasks. TL can improve employees' PE perception and stimulate EIB. Vandenberghe [38] also pointed out that PE is an important mediating variable in the impact of TL on organizational citizenship behavior
3. The EU positively moderates the relationship between TL and PE; that is, the interaction between EU and TL positively affects employees' PE. Based on the above research conclusions, it can be further inferred that the EU positively regulates the mediating role of PE in the relationship between TL and EIB. This finding expands the boundary conditions for TL to stimulate EIB and confirms that TL can stimulate EIB through the mediating role of PE in a high uncertainty environment

Based on the UIT, when employees perceive high and long-term uncertainty, employees will have strong anxiety, prompting employees to urgently obtain organizational identity and self-identity classification and confirmation. Driven by this, employees will independently identify with organizations or groups with the same or similar values, thereby reducing uncertainty by providing oneself with an effective identity that can describe and define “who I am” and “how I should do” [10].

RETRACTED

TL is good at transforming the EU into opportunities and challenges. TL also influences subordinates to internalize organizational goals at the psychological level, forming a unified organizational value and cultural atmosphere, which is conducive to promoting employees' sense of belonging, forming a fault-tolerant organizational environment and innovative organizational support atmosphere, and further increasing employees' recognition of the organization. Based on the perspective of social exchange, employees will reward the organization through innovative behavior practices that benefit the organization. Hogg et al. [23] also confirmed that under high uncertainty, the individual's recognition of the group increases with the increase of group entity, and this entity organization has a homogeneous ideology. Under low uncertainty, identity is not affected by group entitativity.

### 6.2. Management Implications

First, from the perspective of entrepreneurship, TL can stimulate EIB through PE in a high uncertainty environment. This enlightens people that when the uncertainty of the internal and external environment is high, enterprises can stimulate EIB through the influence of TL behavior and PE. On the one hand, it is required that enterprise leaders should have the quality and behavior characteristics of TL. Enterprise managers should cultivate TL style, TL thinking, and cognitive ability. Enterprises can train and audit managers' TL style. Leaders should self-examine and self-improve TL's ability and constantly improve leadership behavior.

On the other hand, based on the innovative characteristics of entrepreneurship, leaders should consciously improve employees' perception of empowerment, create a good atmosphere of empowerment, and respect and trust employees. For example, when assigning challenging work tasks to competent employees, it is necessary to clarify work objectives and inform employees of the importance of work, fully trust and empower employees, and give employees full autonomy, so that employees have higher autonomy and self-efficacy. Employees feel respected and trusted by the organization. Based on reciprocal responsibilities, employees will practice more innovative behaviors that are beneficial to the organization.

Second, in the current era of environmental change, environmental response speed and EU management capabilities become necessary abilities for the CEO. Enterprise leaders should pay more attention to changes in the external environment, quickly perceive changes in the needs of the market and customers, constantly adjust the organizational structure and organizational behavior, and set reasonable organizational goals. Through reasonable incentives and personal support, employees can internalize organizational goals, and create a unified value of organizational culture to enhance employee recognition of the organization.

In addition, in an uncertain environment, while encouraging and guiding employees to participate in organizational change and innovation, people should also pay attention to caring for employees' emotional attribution needs, create an inclusive organizational culture atmosphere, improve employees' psychological safety at work, and create a fair and trusted organizational atmosphere to reduce employees' uncertain perception of the working environment. Therefore, it can reduce the pressure and threats that EIB may face, prompt employees to focus more on their work, and stimulate EIB.

RETRACTED

## 7. Conclusions and Prospects

Through the study of the process of employees' PE to stimulate EIB and in an uncertain environment, based on the perspective of entrepreneurship, a theoretical analysis of the management of stimulating EIB is made, and the relationship between TL and EIB is studied. The results show that the EU has a positive moderating effect on the relationship between TL and PE, while PE positively promotes EIB. The indirect effects of PE from low to high are 0.2221, 0.3495, and 0.4450, respectively. The innovation is to study the scheme of managing EIB based on entrepreneurship in an uncertain environment.

The limitations include the following: First, the concept of EU is often used in research at the strategic level of an organization, but it is rarely used in research on individual relationships. Based on the perspective of UIT, the moderating effect of EU on TL and PE is explored, and then, the influence mechanism of TL on EIB under an uncertain environment is studied. In the future, what kind of leadership behavior can effectively stimulate EIB in an uncertain environment from the perspectives of interdependence theory and social cognitive theory can be further explored. Second, cross-sectional data is used, and the samples are mainly from enterprises in the Chinese context. The relatively insufficient representation of the samples may affect the rigor and external adaptability of the research conclusions. In the future, longitudinal time series data can be used to obtain research sample data through transnational cross-cultural enterprises to further analyze the causal relationship between variables. Future research will further improve the theoretical structure, expand the sample data set, and get more accurate experimental results.

## Figures and Tables

**Figure 1:** Research model.

**Figure 2:** Research framework.

**Figure 3:** Numerical comparison of psychological empowerment mediation.

**Figure 4:** Mediated regulatory effect numerical comparison results.

**Figure 5:** The moderating effect of EU on the relationship between TL and PE.

**Table 1:** CFA results.

Model	Factor	*χ* ^2^/df	GFI	NFI	TLI	CFI	RMSEA
Four-factor model	A, B, C, D	1.274	0.869	0.885	0.970	0.973	0.031
Three-factor model	A+B, C, D	3.742	0.664	0.659	0.704	0.723	0.098
Two-factor model	A+B+C, D	5.632	0.548	0.481	0.510	0.527	0.127
Single-factor model	A+B+C+D	6.633	0.482	0.388	0.392	0.424	0.141
Judgment value of each index		<2.5	>0.85	>0.85	>0.85	>0.85	<0.08

Note: A, B, C, and D, respectively, represent TL, PE, EU, and EIB; “+” indicates the combination of the two factors.

RETRACTED

**Table 2:** Descriptive statistics and Pearson correlation of research variables.

Variable	*M*	SD	1	2	3	4	5	6	7	8
(1) Gender	1.32	0.47	1							
(2) Age	1.52	0.56	0.02	1						
(3) Education level	3.62	0.68	0.66	0.03	1					
(4) Working seniority	2.87	0.97	0.03	0.21	0.24	1				
(5) TL	3.38	0.69	-0.02	-0.14	0.34^∗^	0.17^∗^	1			
(6) PE	2.88	0.64	-0.11	0.16	-0.06	-0.02	0.57^∗∗^	1		
(7) EIB	3.32	0.98	0.04	-0.07	0.18	0.16	0.44^∗∗^	0.59^∗∗^	1	
(8) EU	2.84	1.07	-0.08^∗^	-0.23	-0.07	0.09	-0.02	0.15^∗^	0.01	1

Note: sample size *N* = 287; ∗∗ indicates *p* < 0.01, and ∗ denotes *p* < 0.05.

**Table 3:** Hypothesis test results by hierarchical regression analysis.

Variable	PE			EIB		
Model	Model 1	Model 2	Model 3	Model 4	Model 5	Model 6
Control variable						
Gender	-0.015	-0.041	-0.042	0.081	0.073	0.088
Age	0.016^∗^	0.016	0.018	-0.077	-0.053	-0.085
Educational level	-0.037	-0.018	-0.008	-0.056	-0.025	-0.037
Working seniority	0.045	0.043	0.040	0.052	0.030	0.030
Independent variable						
TL	0.599^∗∗∗^	0.561^∗∗∗^	0.454^∗∗^	0.471^∗∗∗^		0.191^∗∗∗^
Mediating variable						
PE					0.601^∗∗∗^	0.500^∗∗∗^
Moderating variable						
EU		0.164^∗∗^	0.148^∗∗^			
Interactive item: TL∗EU			0.363^∗∗^			
*R* ^2^	0.322	0.348	0.364	0.210	0.356	0.380
*F*	26.732^∗∗∗^	24.894^∗∗∗^	22.788^∗∗∗^	14.964^∗∗∗^	31.077^∗∗^	28.554^∗∗∗^
Δ*R*^2^	0.286	0.026	0.016	0.203	0.349	0.169
Δ*F*	118.658^∗∗∗^	10.963^∗∗^	6.968^∗∗^	72.163^∗∗∗^	152.127^∗∗∗^	76.423^∗∗∗^

Note: ∗∗∗ means *p* < 0.001; ∗∗ refers to *p* < 0.01; ∗ indicates *p* < 0.01.

**Table 4:** Bootstrap test results of PE mediation.

Effect	*β*	Boot SE	LLCI	ULCI	*p*
Direct effect (*C*′)	0.2249	0.0823	0.0629	0.3870	0.0067
Indirect effect (*a*∗*b*)	0.4051	0.0573	0.2955	0.5188	0.0000

**Table 5:** Test results of the mediated regulatory effect.

Mediating variable	Moderating variable	Direct effect (*β*)	Boot SE	LLCI	ULCI
PE	EU (low)	0.2221	0.0739	0.766	0.3690
	EU (medium)	0.3495	0.0540	0.2472	0.4600
	EU (high)	0.4450	0.0627	0.3240	0.5694

## Data Availability

The data used to support the findings of this study are included within the article.
